# Another Way to Perform a Pediatric MRI Avoiding Sedation After Hours When Anesthesia Is Less Accessible: The Skin-to-Skin Technique

**DOI:** 10.7759/cureus.46929

**Published:** 2023-10-12

**Authors:** Tom Saliba, Grammatina Boitsios

**Affiliations:** 1 Radiology, Hôpital Universitaire des Enfants Reine Fabiola, Brussels, BEL; 2 Pediatric Neuroradiology, Hôpital Universitaire des Enfants Reine Fabiola, Brussels, BEL

**Keywords:** anaesthesia, sedation, pediatric, mri, pediatric mri

## Abstract

This innovative system for conducting pediatric MRI describes a method of calming children by allowing them to rest on their accompanying adult's abdomen during the examination. This approach reduces their agitation, enabling the acquisition of diagnostic images when anesthesia is either unavailable or not advisable.

## Introduction

It is widely recognized that the quality of pediatric MRI examinations depends significantly on the patient's cooperation. Severe distress in children can result in the premature termination of exams, as previous studies have indicated [1,2]. Several techniques for calming children during exams exist, including animal-assisted therapy, creating a child-friendly environment, and providing distraction through videos. However, these methods often have drawbacks, such as being time-consuming, expensive, and frequently unavailable [3]. Furthermore, not all of these approaches are suitable for MRI exams, making the need for alternative solutions apparent.

Furthermore, it is generally agreed that children from around six months of age to five years of age, as well as older children with mental disabilities, will require sedation for an MRI exam [3]. However, it is not uncommon to have children within that age range for whom sedation cannot be performed for medical reasons as well as a lack of available anesthetists [3].

When this happens, we are often confronted with exams that either cannot go ahead due to the patient’s unwillingness to enter the machine or children who are coerced into entering the machine but are unable to be still enough to have an examination of diagnostic quality.

## Technical report

This new method was employed in the case of a three-year-old boy who presented to the emergency department with fever, an inflammatory syndrome, and right iliac fossa pain. The clinician referred the patient to the radiology department for suspected appendicitis. The initial ultrasound was non-contributory, with the appendix not being visualizable. Furthermore, due to the age of the patient, the little intra-abdominal fat would likely have made him a poor candidate for an abdominal CT scan due to the difficulty in discerning the different intestinal loops. This exam also required contrast and therefore has been more invasive. Furthermore, an MRI is preferable to a CT scan due to the fact that it is non-irradiating and that a higher radiation dosage may be necessary to have the required contrast for the abdominal exam.

To visualize the appendix while avoiding using an irradiating and contrast-enhanced examination method, an abdominal MRI was proposed by the radiologist. In preparation for the abdominal 1.5 T MRI, the procedure was explained to the mother, who in turn explained the steps to her child to calm them.

Despite much time and effort to attempt to get the child to accept the MRI exam, the child refused to lie on the magnetic resonance examination table for the duration of the examination time, being extremely agitated and thwarting any attempt at a diagnostic exam. We, therefore, suggested to the mother, who was accompanying the child, to lie down in the MRI herself (after checking that she had no contraindication for doing so) and lay her son on top of her, abdomen to abdomen. This compromise was acceptable to the child, who was sufficiently calmed and reassured, agreeing to the examination and entering the machine. The child proceeded to lie on his mother’s abdomen; headphones were placed over the ears of the mother and child to protect them from the noise level of the MRI, and ventilation within the scanner was activated for more comfort.

The rapid examination protocol was carried out, and the examination was of diagnostic quality, allowing the exclusion of any significant intra-abdominal pathology as well as resulting in the detection of a pulmonary infection that had hitherto gone unnoticed (Figures 1-4).

**Figure 1:** 1.5 T MRI axial scout image with a relatively large field of view showing the child atop his mother’s abdomen.

**Figure 2:** 1.5 T MRI T2-weighted axial imaging of the same child’s abdomen demonstrating that images of diagnostic quality are achievable using our abdomen-to-abdomen method.

**Figure 3:** Another 1.5 T MRI T2-weighted coronal imaging of the same child’s abdomen demonstrating the quality of coronal imaging using the abdomen-to-abdomen method.

**Figure 4:** 1.5 T MRI T2-weighted sagittal imaging of the same child’s abdomen and spine, with the incidental finding of a pulmonary lesion (arrow).

Description of method

The abdomen-to-abdomen positioning method is a simple way of attempting to calm children sufficiently to be able to perform an MRI exam of diagnostic quality.

It consists of laying the parents or guardian of the child face up in the MRI scanner and then laying the child, abdomen to abdomen, on top of them. Care must be taken that both the child and adult fit comfortably within the limited space of the MRI and that the coil can be placed in a way that it will not slide off the back of the child. Ear protection is fitted to the adult and child before they are put into the machine. The parent is then instructed to hold the child and the restraining straps are placed around the adult and the child to hold them in place. Verbal instructions are given to both the adult and child to remain still throughout the exam. The emergency button is handed to the adult, who is instructed to activate it if they or the child begins to experience any unreasonable amounts of discomfort. With this setup, we were able to achieve images of similar quality to what we would expect to have in children of similar size and weight who entered the MRI alone.

Given the unpredictable nature of this method, we recommend starting with essential and preferably quick MRI sequences before considering non-essential ones. Our full protocol is performed in about 10 minutes, consisting of three T2 haste weighted sequences in each orthogonal axis requiring 20 seconds each, a T1-weighted vibe Dixon sequence requiring 15 seconds, an axial T2-weighted sequence with fat suppression requiring 40 seconds, and an axial diffusion-weighted sequence requiring 60 seconds. We believe that performing an exam with contrast is technically feasible in this configuration, though thus far, we have made no attempt to do so as we have not encountered a situation requiring it in which this technique has been used.

Although the above example was performed for abdominal imaging, we have also performed a slightly modified procedure for a brain MRI in which the mother laid next to the two-and-a-half-year-old child whose head was encased in the coil.

## Discussion

This method’s main advantage can be easily summarized. It allows imaging of reasonable quality in children that would otherwise have been deemed impossible and resulted in the cancellation of the exam. In cases where the children are uncooperative, the acquired images are often of non-diagnostic quality, making sedation necessary for the exam to be successful. This method should be used to gain the images essential for a diagnosis without needlessly prolonging the exam or requiring sedation.

Despite the usefulness of this method, there are, unfortunately, some drawbacks. One should exercise caution in cases where this approach may not be feasible, such as when the adult is pregnant, has a non-MRI compatible or metallic implant, suffers from claustrophobia, or has a body habitus that may cause the child to slip off their abdomen if not properly secured.

The radiologist must also perform the mental gymnastics necessary to correctly interpret the image if the child is in an unusual position, such as being prone or laid on their side, which may cause changes compared to dorsal decubitus images such as the relative positions of gas and fluids under the effect of gravity.

Furthermore, we do not have any data regarding the possible issues related to the specific absorption rate caused by having a much larger adult in the same field as a child, though their larger relative body surface area may be advantageous for dissipating heat [4]. We also do not have any data on possible issues regarding the signal-to-noise ratio, which will require further study.

We do not specifically believe that this method should be limited to the mother but to any adult the child feels comfortable with and does not have any of the aforementioned contraindications.

## Conclusions

In conclusion, while this method may serve as a last resort when all other options have been exhausted and the examination must proceed urgently, it should not be chosen when more effective methods, such as pediatric anesthesia, are available or considered appropriate. Nevertheless, we believe that this method merits further investigation, as it may offer a solution in otherwise challenging cases where anesthesia is not a viable option or in cases of patients with semi-urgent conditions who are not ideal MRI patients.
